# Gasdermin D Deficiency Does Not Protect Mice from High-Fat Diet-Induced Glucose Intolerance and Adipose Tissue Inflammation

**DOI:** 10.1155/2022/7853482

**Published:** 2022-08-26

**Authors:** Eun Bi Ma, Hafiz Muhammad Ahmad Javaid, Do-Hyeon Jung, Jong-Hwan Park, Joo Young Huh

**Affiliations:** ^1^College of Pharmacy, Chonnam National University, Gwangju, Republic of Korea; ^2^Laboratory Animal Medicine, College of Veterinary Medicine, Chonnam National University, Gwangju, Republic of Korea

## Abstract

The adipose tissue NLRP3 inflammasome has recently emerged as a contributor to obesity-related metabolic inflammation. Recent studies have demonstrated that the activation of the NLRP3 inflammasome cleaves gasdermin D (GSDMD) and induces pyroptosis, a proinflammatory programmed cell death. However, whether GSDMD is involved in the regulation of adipose tissue function and the development of obesity-induced metabolic disease remains unknown. The aim of the present study was to investigate the role of GSDMD in adipose tissue inflammation as well as whole-body metabolism using GSDMD-deficient mice fed a high-fat diet (HFD) for 30 weeks. The effects of GSDMD deficiency on adipose tissue, liver, and isolated macrophages from wild-type (WT) and GSDMD knockout (KO) mice were examined. In addition, 3T3-L1 cells were used to examine the expression of GSDMD during adipogenesis. The results demonstrate that although HFD-induced inflammation was partly ameliorated in isolated macrophages and liver, adipose tissue remained unaffected by GSDMD deficiency. Compared with the WT HFD mice, GSDMD KO HFD mice exhibited a mild increase in HFD-induced glucose intolerance with increased systemic and adipose tissue IL-1*β* levels. Interestingly, GSDMD deficiency caused accumulation of fat mass when challenged with HFD, partly by suppressing the expression of peroxisome proliferator-activated receptor gamma (PPAR*γ*). The expression of GSDMD mRNA and protein was dramatically suppressed during adipocyte differentiation and was inversely correlated with PPAR*γ* expression. Together, these findings indicate that GSDMD is not a prerequisite for HFD-induced adipose tissue inflammation and suggest a noncanonical function of GSDMD in regulation of fat mass through PPAR*γ*.

## 1. Introduction

Obesity has emerged as a global epidemic as it has increased the incidence of several metabolic disorders, such as type 2 diabetes, nonalcoholic fatty liver disease (NAFLD), and atherosclerosis [1]. Among several factors responsible for the pathogenesis of obesity, recent studies have emphasized the role of sterile inflammation of adipose tissue in the development of obesity-related metabolic disorders [2, 3]. In response to caloric excess, adipocyte hypertrophy leads to the infiltration of immune cells such as macrophages, resulting in the secretion of inflammatory cytokines from adipose tissue [4, 5]. Moreover, adipocytes can synthesize and secrete proinflammatory adipokines to induce inflammation and insulin resistance in adipocytes as well as recruit macrophages to further infiltrate adipose tissues [6, 7]. Therefore, adipose tissue is considered an active immunological organ, and dysfunctional adipose tissue with low-grade, chronic inflammation is linked to the pathogenesis of obesity-related metabolic diseases [2, 8].

The adipose tissue NLRP3 inflammasome has recently emerged as a contributor to obesity-related metabolic inflammation [9]. Excessive saturated fatty acids and reactive oxygen species in hypertrophic adipocytes can activate the NLRP3 inflammasome and subsequently cleave caspase-1, which in turn converts pro-interleukin- (IL-) 1*β*/pro-IL-18 into functional IL-1*β*/IL-18 [9]. Studies have demonstrated that caspase-1 can also cleave gasdermin D (GSDMD) and induce pyroptosis [10]. The cleaved gasdermin-N domain (GSDMD-N) oligomerizes to form pores in the cell membrane, thus mediating the release of IL-1*β*/IL-18 or inducing cell death by rupturing the membrane [11]. Pyroptosis therefore represents a typical proinflammatory programmed cell death process, which can promote the development of various diseases, including nonalcoholic steatohepatitis (NASH) and diabetic nephropathy [12, 13]. In hypertrophic adipocytes, Giordano et al. reported that NLRP3-dependent caspase-1 activation triggers pyroptosis [14]. However, the potential role of GSDMD in adipose tissue and the underlying mechanism in obesity remain unknown. Therefore, understanding the mechanism governing the role of GSDMD in obesity will assist in understanding low-level adipose tissue inflammation and provide new ideas for developing therapeutics against obesity and related metabolic diseases.

In the present study, we investigated whether GSDMD is involved in the regulation of adipose tissue function and the development of obesity-induced metabolic disease using GSDMD-deficient mice. Our results demonstrate that although high-fat diet- (HFD-) induced inflammation is partly ameliorated in isolated macrophages and liver, adipose tissue is not affected by GSDMD deficiency. Moreover, GSDMD deficiency causes a mild increase in glucose intolerance and adiposity when challenged with a HFD, partly by regulating the expression of peroxisome proliferator-activated receptor gamma (PPAR*γ*). These findings provide insights into the function of GSDMD in adipose tissue and the mechanism underlying inflammation in the pathophysiology of obesity.

## 2. Materials and Methods

### 2.1. Animal Studies

Wild type (WT) mice on a C57BL/6 background were purchased from Jackson Laboratory (Bar Harbor, ME, USA). GSDMD knockout (KO) mice were kindly provided by Gabriel Núñez (University of Michigan Medical School, Ann Arbor, MI, USA). All mice were housed in a pathogen-free animal facility at 22 ± 2°C and a humidity of 55 ± 5%, under a 12 h light/12 h dark cycle. Eight-week-old WT and GSDMD KO mice were randomly divided into two groups: those fed a normal chow diet (NCD) and those fed a HFD, respectively. The NCD mice were fed a standard diet composed of 4.5% fat (3.41 kcal/g), whereas HFD mice were fed a diet containing 60% fat, 21.3% carbohydrate, and 18.4% protein (5.24 kcal/g, Research Diets, Inc., New Brunswick, NJ, USA). All mice were provided food and water *ad libitum*. All animal studies were approved by the Institutional Animal Care and Use Committee at the Chonnam National University.

### 2.2. Glucose and Insulin Tolerance Test

An oral glucose tolerance test (OGTT) was performed after mice were fasted overnight for 12 h. Glucose (D-glucose) was administered by oral injection at a dose of 2 g glucose/kg body weight. The level of glucose in the blood was measured 0, 15, 30, 60, 120, and 180 min after glucose injection. An intraperitoneal insulin tolerance test (IPITT) was performed after overnight fasting for 6 h. Insulin (Sigma; St. Louis, MO, USA) was administered intraperitoneally (1 U/kg of body weight). Blood glucose levels were measured at 0, 15, 30, 60, and 120 min after insulin injection.

### 2.3. Cell Culture

3T3-L1 mouse preadipocytes were purchased from the American Type Culture Collection (Manassas, VA, USA). The cells were maintained in Dulbecco's modified Eagle medium with 10% fetal bovine serum (HyClone, Australia) and 1% penicillin/streptomycin (Carlsbad, CA, USA) and incubated at 37°C in 5% CO_2_. Two days after 100% confluency (day 0), the 3T3-L1 cells were treated with 1 *μ*g/mL insulin (Sigma), 0.25 *μ*M dexamethasone (Sigma), and 0.5 mM 1-methyl-3-isobutylxanthine (Sigma) and 1 *μ*M rosiglitazone (Sigma) in DMEM supplemented with 10% FBS and 1% penicillin/streptomycin. After 2 days, differentiation medium was replaced with 1 *μ*g/mL insulin and DMEM supplemented with 10% FBS and 1% penicillin/streptomycin. Thereafter, the medium was replaced with a medium containing 10% FBS every 48 h until day 6.

### 2.4. Primary Murine Bone Marrow-Derived Macrophage (BMDM) Culture

Mice were sacrificed via cervical dislocation. Bone marrow cells were collected from the tibia and fibula. After centrifuging at 10,000 rpm for 1 min, cells were seeded into cell culture plates and incubated at 37°C for 7 days using Iscove's Modified Dulbecco's Medium (Gibco, Carlsbad, CA, United States) supplemented with 10% FBS, 30% L929-conditioned media, 1% penicillin/streptomycin, 1% sodium pyruvate, and 1% MEM nonessential amino acids. BMDMs were primed for 6 h with 100 ng/mL lipopolysaccharide (LPS, Sigma), followed by 2 mM ATP (Sigma) treatment for the final 30 min before harvesting.

### 2.5. Gene Expression Analysis

The total RNA was isolated from the liver, visceral, and subcutaneous adipose tissue using TRIzol (MRC, Cincinnati, OH, USA) and reverse-transcribed into complementary DNA (cDNA) by TOPscript™ RT DryMIX (Enzynomics, South Korea). A quantitative real-time polymerase chain reaction (PCR) was performed using the TOPreal SYBR Green PCR Kit (Enzynomics). The mRNA levels were detected by real-time PCR using the Rotor-Gene Q PCR cycler (QIAGEN, Hilden, Germany). The level of mRNA was normalized to 18S ribosomal RNA.

### 2.6. Western Blotting

Tissue lysates and 3T3-L1 cells were homogenized with RIPA buffer (Thermo Scientific, Rockford, IL, United States). Protein concentration was determined using the Pierce BCA Protein Assay Kit (Thermo Fisher Scientific). Western blotting was performed as described previously [15]. Anti-GSDMD (ab219800) antibody was purchased from Abcam (Cambridge, UK), and anti-adiponectin (AG-20A-0003) antibody was procured from AdipoGen (Seoul, Korea). Anti-Bax (#14796), anti-GPX4 (#59735), and anti-*β*-tubulin (#2146) antibodies were purchased from Cell Signaling Technology (Danvers, MA), and anti-caspase-1 (sc-56036) and anti-*β*-actin (sc-47778) antibodies were purchased from Santa Cruz Biotechnology, Inc. (Dallas, TX, USA).

### 2.7. Enzyme-Linked Immunosorbent Assay (ELISA)

Protein levels of IL-1*β* and IL-18 were measured using ELISA kits. The IL-1*β* levels in the liver, adipose tissue, and plasma were measured using commercial ELISA kits purchased from Invitrogen (Carlsbad, CA, USA) according to the manufacturer's instructions. The levels of IL-18 in the plasma were determined using the ELISA kit purchased from MBL Life Science (Nagoya, Japan).

### 2.8. GSH Detection Assay

Liver and VAT samples were measured using a GSH/GSSG Ratio Detection Assay Kit (#ab205811; Abcam) according to the manufacturer's instructions. Fluorescence was monitored at 490/520 nm using a Synergy HTX Multimode Microplate Reader (Agilent, Santa Clara, USA).

### 2.9. Statistics

All statistical analyses were conducted using StatView v5.0 software (SAS Institute, Inc., Cary, NC, USA). Graphs were constructed with GraphPad Prism. All results are presented as the mean ± standard error of the mean. One-way analysis of variance (ANOVA) was performed to compare mean values between groups, followed by Fisher's protected least significant difference (PLSD) *post hoc* test. Associations between GSDMD and PPAR*γ* were assessed with Pearson's correlation coefficient. *P* values less than 0.05 were considered to be statistically significant.

## 3. Results

### 3.1. Gasdermin D Deficiency Promotes HFD-Induced Adipose Tissue Accumulation without Change in Body Weight

We first examined whether a deficiency in GSDMD could influence the development of obesity in mice fed NCD or HFD for 30 weeks. The mice in the WT HFD group showed significantly elevated weight gain compared to those in the WT NCD group (Figures 1(a) and 1(b)). The weight gain in GSDMD KO mice was comparable to that observed in WT mice, with no significant changes in food consumption among the groups on the same diet (Figures 1(c) and 1(d)). Despite no differences in body weight, subcutaneous adipose tissue and visceral adipose tissue (VAT) weight was significantly increased in GSDMD KO HFD mice compared with WT HFD mice (Figures 1(e) and 1(f)). These differences remained significant after adjusting for body weight. Liver weight was also increased by HFD; however, the increase was comparable between WT and GSDMD KO mice (Figure 1(g)). These findings indicate increased adiposity in GSDMD KO mice without any change in body weight.

### 3.2. Gasdermin D Deficiency Induces a Mild Increase in Glucose and Insulin Intolerance

Since obesity is associated with the development of insulin resistance, we next determined the effect of HFD on glucose and insulin tolerance in WT and GSDMD KO mice. At 15 weeks on HFD, impairments in glucose tolerance were observed compared to mice fed a NCD, independent of phenotype (Figure 2(a)). After 30 weeks on HFD, no impairments were observed in WT mice, whereas the increase in the area under the curve (AUC) remained significant in GSDMD KO mice fed HFD compared to those fed NCD (Figure 2(c)). The less pronounced differences observed in WT mice imply that mice fed NCD became glucose intolerant over time. The IPITT results showed impairments in WT mice at both 15 and 30 weeks on HFD compared to NCD-fed mice (Figures 2(b) and 2(d)). Compared with WT HFD mice, the AUC was significantly larger in GSDMD KO HFD mice at 15 weeks but not at 30 weeks. These results imply that along with increased adiposity, deficiency in GSDMD does not protect against HFD-induced metabolic impairments, but that it rather prompts a mild glucose and insulin intolerance.

Because GSDMD is involved in the formation of membrane pores and the secretion of proinflammatory cytokines [11], we next assessed the levels of IL-1*β* and IL-18 in the plasma. Although WT mice fed HFD did not show elevated plasma IL-1*β* levels, an unexpected increase in IL-1*β* levels was observed in GSDMD KO HFD mice compared with WT HFD mice (Figure 2(e)). In contrast, compared with those observed in WT NCD mice, IL-18 levels were downregulated in GSDMD NCD mice and further decreased in GSDMD HFD mice, although the decrease was not statistically significant (Figure 2(f)). Altogether, these results indicate that GSDMD deficiency causes a mild increase in HFD-induced glucose and insulin tolerance along with upregulated IL-1*β* levels.

### 3.3. Gasdermin D Deficiency Inhibits HFD-Induced Inflammation in the Liver without Any Change in Metabolism

Previous studies have demonstrated that GSDMD functions as a pyroptosis executor of NASH, and GSDMD KO mice fed a methionine-choline deficient (MCD) diet showed reduced steatohepatitis compared with WT mice [12, 16]. Therefore, we sought to examine the inflammatory and metabolic response to HFD in the GSDMD KO mouse liver. We first confirmed the levels of GSDMD protein in the liver and showed that neither full-length nor cleaved forms of GSDMD were detected in GSDMD KO mice (Figure 3(a)). Accordingly, liver IL-1*β* protein levels showed a decreasing trend in GSDMD KO HFD mice compared with the levels observed in WT HFD mice (Figure 3(b)). The expression of caspase-1 protein was lower in HFD mice compared to NCD mice, independent of genotype (Figure 3(c)).

The expression of inflammatory genes showed that HFD induced the expression of GSDMD, IL-1*β*, and monocyte chemoattractant protein-1 (MCP-1) mRNAs in WT mice compared to NCD-fed mice (Figure 3(d)). In GSDMD-deficient HFD mice, the mRNA expression of tumor necrosis factor alpha (TNF*α*) and MCP-1 was significantly decreased compared to that observed in WT HFD mice. The mRNA expression of IL-1*β* and IL-18 also exhibited a diminishing trend in GSDMD KO HFD mice compared to that seen in WT HFD mice, although the difference was insignificant. In addition, we examined the markers of autophagy, which is known as an upstream regulator of pyroptosis [17]. The results were similar to those for markers of inflammation in that HFD-induced p62 and ATG7 mRNA expressions in WT mice were suppressed in GSDMD KO mice (Figure 3(f)). Studies have reported a relationship between pyroptosis and other cell death pathways, including apoptosis [18, 19] and ferroptosis [20]. Therefore, we examined whether these pathways are regulated by GSDMD in the liver. While markers of apoptosis (Bax, caspase-9, and Bcl-2) were significantly increased in WT HFD mice compared to WT NCD mice, only Bax mRNA expression was reversed in GSDMD KO HFD mice (Figure 3(e)). Decreased glutathione peroxidase 4 (GPX4) and glutathione (GSH) expressions imply ferroptosis induction [21, 22]. While GPX4 mRNA expression was increased in our HFD-fed GSDMD KO mice compared to the NCD mice, GSH levels were significantly decreased in the HFD-fed GSDMD KO mice compared to both WT HFD and NCD-fed GSDMD KO mice, implying increased vulnerability towards oxidative stress [23].

Next, we evaluated whether the amelioration of inflammation by GSDMD deficiency led to changes in liver metabolism. The expression of mitochondrial genes (PRX3, PGC1*α*, and CPT1*α*) and lipolysis genes (ATGL and HSL) was examined (Figures 3(g) and 3(h)). While PRX3, CPT1*α*, and HSL mRNA expressions were significantly elevated by HFD in WT mice, only PRX3 mRNA expression was downregulated by GSDMD deficiency. These results imply that although a deficiency in GSDMD partly reverses HFD-induced hepatic inflammation, it does not lead to the regulation of metabolism in the liver.

### 3.4. Gasdermin D Deficiency Exerts No Effect on HFD-Induced Adipose Tissue Inflammation

While there are recent reports on the role of GSDMD in the liver, the effect of GSDMD in adipose tissue remains unidentified. We therefore examined the effect of GSDMD deficiency on adipose tissue inflammation and metabolism. In contrast to our results in the liver, HFD-induced mRNA expression of NLRP3, IL-18, IL-6, and MCP-1 in the VAT of WT mice was not suppressed by GSDMD deficiency (Figure 4(a)). Interestingly, NCD-fed GSDMD KO mice exhibited elevated levels of TNF*α* and IL-6 mRNA compared to WT NCD mice. Moreover, the mRNA and protein expressions of IL-1*β* in adipose tissue were elevated in GSDMD KO HFD mice compared to that seen in WT HFD mice (Figure 4(b)), which is in line with the elevated plasma levels of IL-1*β* observed in GSDMD KO HFD mice. HFD-induced p62 mRNA expression in WT mice was reversed in HFD-fed GSDMD KO mice, while ATG7 was unaltered in any of the groups (Figure 4(c)). Next, we examined whether apoptosis and ferroptosis were affected by GSDMD deficiency in adipose tissue. As shown in Figures 4(d) and 4(e), the expression of Bax and Bcl-2 was significantly upregulated in WT HFD mice compared to WT NCD mice. While Bax mRNA and protein levels were suppressed in GSDMD KO HFD mice, Bcl-2 mRNA remained unchanged compared to the levels observed in WT HFD mice. GPX4 mRNA and protein levels were unaffected by GSDMD deficiency in adipose tissue (Figures 4(d) and 4(f)); however, GSH levels were elevated in GSDMD KO mice, suggesting a compensatory increase due to the elevation of inflammation in GSDMD KO mice. Next, we measured the effect of GSDMD deficiency on the expression of metabolic genes. Similar to the changes seen in inflammatory genes, the mRNA expression of leptin, adiponectin, resistin, PGC1*α*, and CPT1*α* was significantly elevated in WT HFD mice, comparable to the elevation observed in GSDMD KO HFD mice (Figures 4(g) and 4(i)). The protein levels of adiponectin remained unaltered in all groups (Figure 4(j)). Altogether, these data suggest that a lack of GSDMD does not ameliorate inflammation or metabolic dysfunction of adipose tissue.

### 3.5. Gasdermin D Deficiency Regulates ATGL and PPAR*γ* Expression in Adipose Tissue

Adipose tissue mass is determined by the amount of stored and removed triglycerides in adipocytes as well as adipocyte differentiation [24]. Because we observed a significant increase in the fat mass of GSDMD KO HFD mice compared with WT HFD mice, we next studied the mechanism responsible for this phenomenon. ATGL and HSL are key enzymes involved in the intracellular degradation of triglycerides [25, 26]. Our results showed that although the mRNA levels of ATGL and HSL were increased in WT mice in response to a HFD, their expression levels were suppressed in GSDMD KO HFD mice, indicating a decrease in lipolysis (Figure 4(h)). In addition, the expression of PPAR*γ* mRNA and protein was significantly suppressed in both NCD- and HFD-fed GSDMD KO mice compared to WT mice (Figures 5(a) and 5(b)). PPAR*γ* is a central regulator of lipid metabolism; it performs this function by regulating lipid uptake and adipocyte differentiation [27]. Adipogenesis through PPAR*γ* activation supports healthy adipose tissue remodeling in obesity [28, 29]. To examine whether GSDMD is related to adipocyte differentiation, its levels were monitored during 3T3-L1 adipocyte differentiation. PPAR*γ* mRNA levels were increased during adipogenesis as expected (Figure 5(c)). As shown in Figures 5(d) and 5(e), the levels of GSDMD mRNA and protein significantly decreased in a time-dependent manner during adipogenesis. Moreover, the correlation analysis between PPAR*γ* and GSDMD genes showed a negative correlation (Figure 5(f)). These results reveal the possibility of a noncanonical role of GSDMD in regulating adipogenesis, which may lead to the regulation of adipose tissue remodeling.

### 3.6. Gasdermin D Deficiency Attenuates HFD-Induced Macrophage Activation

Previous studies have demonstrated that the infiltration of macrophages into adipose tissue is the primary source of NLRP3 inflammasome activation in obesity [30, 31]. To elucidate the effect of GSDMD deficiency on macrophage activation, we isolated BMDMs from WT and GSDMD KO mice fed NCD or HFD and stimulated macrophage activation by treatment with LPS and ATP. First, low expression of GSDMD mRNA was confirmed in NCD- and HFD-fed GSDMD KO mice macrophages compared to WT mice macrophages (Figure 6(a)). Compared with WT NCD macrophages, macrophages isolated from WT HFD mice showed elevated expression of NLRP3 and GSDMD mRNA and IL-1*β* secretion after stimulation (Figures 6(a), 6(b), and 6(d)). Despite their GSDMD deficiency, the expression of NLRP3 mRNA was elevated in both GSDMD NCD and HFD macrophages after treatment with LPS (Figure 6(b)). Although the expression of IL-1*β* mRNA was significantly inhibited in macrophages isolated from both NCD- and HFD-fed GSDMD KO mice compared with those isolated from the WT group (Figure 6(c)), the secretion of IL-1*β* decreased in the GSDMD KO HFD macrophages compared with that in WT HFD macrophages, but not in the GSDMD KO NCD group (Figure 6(d)). These findings indicate that a lack of GSDMD suppresses the expression of IL-1*β* and secretion in macrophages, which is in contrast to the elevated IL-1*β* expression observed in adipose tissue and the elevated plasma IL-1*β* levels in GSDMD KO mice fed HFD.

## 4. Discussion

GSDMD is a critical effector of pyroptosis, and studies have demonstrated that excessive uncontrolled pyroptosis is implicated in the pathogenesis of metabolic disease [32]. However, the function of GSDMD in adipose tissue has remained elusive. Here, we assessed whether GSDMD is involved in the regulation of adipose tissue inflammation and subsequently in systemic metabolism. Contrary to our expectations, we observed that GSDMD deficiency did not reduce 30 weeks of HFD-induced adipose tissue inflammation. Furthermore, GSDMD KO mice were not protected from HFD-induced systemic glucose and insulin tolerance, compared with WT mice. Interestingly, GSDMD KO mice showed an increase in fat mass, along with a downregulation in the expression of ATGL and PPAR*γ*, implicating a noncanonical role of GSDMD in regulation of fat mass. Altogether, these findings indicate that GSDMD is not required for HFD-induced adipose tissue inflammation, suggesting that other GSDMD-independent mechanisms play a dominant role in mediating adipose tissue inflammation associated with obesity.

To date, the function of GSDMD in metabolism has been most extensively studied in the liver [12, 33, 34]. For instance, Xu et al. reported that hepatic GSDMD-N protein levels were significantly higher in humans suffering from NASH and correlated with the NAFLD activity score and fibrosis and that GSDMD KO mice fed a MCD exhibited decreased severity of steatosis and inflammation compared with WT littermates [12]. Similarly, we observed that HFD-induced inflammatory cytokine expression and secretion were ameliorated by GSDMD deficiency in the liver and BMDMs. However, our OGTT and ITT results showed unaffected or even worsened systemic metabolism in GSDMD KO mice, suggesting the involvement of other tissues in the metabolic dysregulation.

Adipose tissue inflammation is an important determinant of whole-body insulin resistance [3]. Despite the deficiency in GSDMD, HFD-induced expression of adipose tissue inflammatory genes was not suppressed. Moreover, increased expression of IL-1*β* in the adipose tissue was observed in GSDMD KO HFD mice, which was in line with the increased plasma IL-1*β* levels. Recently, an alternative form of lytic cell death was reported in the absence of GSDMD-dependent pyroptosis in cells lacking caspase-1 protease activity, accompanied by a delayed secretion of IL-1*β* that eventually reached equivalent amounts compared to WT cells [35]. Of note, pyroptosis is not the only mechanism required for IL-1*β* secretion; other mechanisms involving exosomes and microvesicles also play a role in the process [36]. Therefore, it is likely that the increase in IL-1*β* observed in our study is due to mechanisms that are independent of GSDMD. In our experiments, IL-1*β* secretion was suppressed in isolated macrophages, indicating that other cell types are involved in increases in circulatory IL-1*β* levels. Interestingly, a recent study discovered that in cell types that do not or only weakly express GSDMD, caspase-1 can induce apoptosis involving the bid–caspase-9–caspase-3 axis, followed by gasdermin E-dependent secondary necrosis/pyroptosis [37]. Our results on apoptotic markers show that while HFD-induced Bax expression was downregulated, Bcl-2 and caspase-9 were unaltered compared to WT HFD mice, implying that deficiency in GSDMD only partially inhibits apoptosis. Ferroptosis is another type of cell death, characterized by a downregulation in GPX4 and GSH levels that leads to lipid peroxidation-mediated cell death [38]. Recent studies have reported that ferroptosis is functionally linked to pyroptosis [39, 40]. In GSDMD KO mice, an opposite pattern of GSH levels was observed in the liver and adipose tissue, with GSH levels decreased in the liver and increased in adipose tissue. This correlates with the contrasting effect of GSDMD deficiency on inflammatory genes in each tissue, suggesting a possible compensatory role of ferroptosis.

Considering that the lack of GSDMD did not abrogate HFD-induced adipose tissue inflammation, it is not surprising that glucose intolerance was not reduced in GSDMD KO mice relative to WT mice. In most studies, NLRP3 and caspase-1 KO mice were found to be resistant to HFD-induced obesity and insulin resistance [41, 42]. However, some have reported contrasting results, with deficiency in NLRP3 and caspase-1 not protecting mice from HFD-induced obesity [43, 44], which suggests that the presence of the NLRP3 and caspase-1 genes is not required for HFD-induced adipose tissue inflammation and glucose intolerance. Surprisingly, these previous studies have observed an increase in adiposity following the loss of the inflammasome gene, which is in line with our observation of an increase in fat mass in GSDMD KO mice. Notably, plasma IL-18 levels were commonly reduced in NLRP3 KO mice [44], caspase-1 KO mice [43], and GSDMD KO mice in our study. Of note, deficiency of IL-18 in mice leads to obesity and insulin resistance, largely due to hyperphagia [45]. However, we did not observe any difference in food intake in GSDMD KO mice, implying that other peripheral roles of IL-18 may have contributed to the accumulation of fat.

Interestingly, we found that the expression of PPAR*γ* was dramatically suppressed in both NCD- and HFD-fed GSDMD KO mice compared with that observed in WT mice. Under physiological conditions, adipocyte death leads to the formation of new adipocytes through adipogenesis [46]. Considering that PPAR*γ* is a master regulator of adipocyte differentiation [27], reduced expression of PPAR*γ* in GSDMD KO mice would block de novo adipogenesis, which may account for the switch in adipose tissue from hyperplasia to hypertrophy. As adipocyte hypertrophy is known as a dominant mechanism of fat cell expansion and enhanced susceptibility to insulin resistance in humans [47], our results imply a noncanonical function of GSDMD in maintaining adipose tissue plasticity through the regulation of PPAR*γ*. Previous reports have shown that PPAR*γ* can interact with NLRP3 [48] and that TNF*α* can induce a caspase-1-mediated degradation of PPAR*γ* in adipocytes [49], but this study is the first to show the link between GSDMD and PPAR*γ*.

Contrary to our hypothesis, GSDMD KO mice were not protected from HFD-induced metabolic dysregulation. One possible explanation for this is differences in diets used across studies. Xu et al. used MCD to induce steatohepatitis [12]. In their study, 4 weeks of MCD diet in control mice or 10 days of a MCD diet in obese *db*/*db* mice significantly induced GSDMD-N expression, while HFD only induced GSDMD-N expression after 36 but not after 11 weeks of diet. Similarly, we failed to observe an increase in total and cleaved GSDMD levels in the liver, which may have caused the differences in phenotype. This can be regarded as a limitation of the current study. Since the discovery of GSDMD as the first key protein involved in pyroptosis through the classical NLRP3–caspase-1 axis, other gasdermins, including gasdermins B, C, and E, have been discovered along with the noncanonical pyroptosis pathway involving caspase-11/4/5 [50]. The existence of other types of gasdermins shows the complexity of the pyroptosis pathway and implies that deficiency in one factor could easily be compensated by other factors.

## 5. Conclusion

Our study demonstrates that although a deficiency in GSDMD suppresses inflammation in the liver and macrophages, adipose tissue inflammation remains unaffected. In addition, a mild increase in fat mass is observed along with inhibited expression of PPAR*γ* in the adipose tissue of GSDMD KO mice fed HFD, implying a novel relationship between GSDMD and adipose tissue remodeling. Since the whole-body knockout of GSDMD exerted a minor effect on metabolism, mechanisms associated with adipose tissue should be studied in adipocyte-specific GSDMD KO mice. Along with the known effect of GSDMD on innate inflammation, our findings provide insights into the function of GSDMD in adipose tissue.

## Figures and Tables

**Figure 1:** Body weight and food intake in wild-type (WT) and gasdermin D knockout (GSDMD KO) mice fed a high-fat diet (HFD). (a and b) Measurements of changes in body weight during a HFD or normal chow diet (NCD) in WT and GSDMD KO mice. (c and d) Measurements of food intake in WT and GSDMD KO mice fed a NCD or HFD. (e–g) Tissue weight and ratio of tissue weight per body weight in subcutaneous adipose tissue (SAT), visceral adipose tissue (VAT), and liver. ^∗^*p* < 0.05 vs. same genotype mice fed a NCD and ^#^*p* < 0.05 vs. WT HFD group.

**Figure 2:** Glucose and insulin tolerance in wild-type (WT) and gasdermin D knockout (GSDMD KO) mice fed a high-fat diet (HFD). (a) Oral glucose tolerance test and (b) intraperitoneal insulin tolerance test performed at 15 weeks on a HFD in WT and GSDMD KO mice. Blood glucose levels were measured and the area under the curve (AUC) was determined. (c) Oral glucose tolerance test and (d) intraperitoneal insulin tolerance test performed at 30 weeks on a HFD in WT and GSDMD KO mice. Plasma IL-1*β* (e) and IL-18 (f) measured by ELISA. ^∗^*p* < 0.05 vs. same genotype mice fed a NCD, ^†^*p* < 0.05 vs. WT NCD group, and ^#^*p* < 0.05 vs. WT HFD group.

**Figure 3:** Liver inflammation and metabolism in wild-type (WT) and gasdermin D knockout (GSDMD KO) mice fed a high-fat diet (HFD). (a) Representative western blots and quantitative analysis of GSDMD in liver. (b) IL-1*β* protein expression in liver was measured by ELISA assay. (c) Representative western blots and quantitative analysis of pro-caspase1 and caspase1 in liver. The expression level of protein was normalized using *β*-tubulin. (d–h) Real-time PCR analysis of genes in the liver. The expression level of each target was normalized using 18S rRNA. (i) GSH concentration in liver was evaluated by GSH Detection Assay kit. ^∗^*p* < 0.05 vs. same genotype mice fed a NCD, ^†^*p* < 0.05 vs. WT NCD group, and ^#^*p* < 0.05 vs. WT HFD group.

**Figure 4:** Adipose tissue inflammation and metabolism in wild-type (WT) and gasdermin D knockout (GSDMD KO) mice fed a high-fat diet (HFD). (a, c, d, g, h, and i) Real-time PCR analysis of genes in visceral adipose tissue (VAT). The expression level of each target was normalized using 18S rRNA. (b) IL-1*β* protein expression in VAT was measured by ELISA assay. (e, f, and j) Representative western blots and quantitative analysis of protein expression in VAT. The protein expression level was normalized using *β*-actin. (k) GSH concentration in VAT was evaluated by GSH Detection Assay kit. ^∗^*p* < 0.05 vs. same genotype mice fed a NCD, ^†^*p* < 0.05 vs. WT NCD group, and ^#^*p* < 0.05 vs. WT HFD group.

**Figure 5:** PPAR*γ* and gasdermin D (GSDMD) expression in 3T3-L1 cells during adipogenesis. (a) Real-time PCR analysis of PPAR*γ* genes in adipose tissue of wild-type (WT) and GSDMD KO mice fed a normal chow diet (NCD) or high-fat diet (HFD). (b) Representative western blot image and quantitative analysis of PPAR*γ* in adipose tissue of WT and GSDMD KO mice. (c and d) Real-time PCR analysis of PPAR*γ* and GSDMD genes during adipogenesis. (e) Representative western blot image and quantitative analysis of GSDMD protein during adipogenesis. Samples were taken before and 2, 4, and 6 days after treatment of 3T3-L1 preadipocytes with differentiation media. (f) Correlation analysis between GSDMD and PPAR*γ* genes during adipogenesis. Protein expression levels were normalized to *β*-actin. Gene expression levels were normalized to 18S rRNA. ^∗^*p* < 0.05 vs. same genotype mice fed a NCD, ^†^*p* < 0.05 vs. WT NCD group, ^#^*p* < 0.05 vs. WT HFD group, and ^ǂ^*p* < 0.05 vs. D+0.

**Figure 6:** Macrophage activation in wild-type (WT) and gasdermin D knockout (GSDMD KO) mice fed a high-fat diet (HFD). (a and c) Bone marrow-derived macrophages were isolated from WT and GSDMD KO mice fed a normal chow diet (NCD) or HFD. Bone marrow-derived macrophages (BMDMs) were treated with LPS, and gene expression of GSDMD and IL-1*β* was measured by real-time PCR. Gene expression levels were normalized to 18S rRNA. (b) Representative western blot image and quantification of NLRP3 after LPS and ATP treatment. Protein expression levels were normalized to *β*-tubulin. (d) Secretion of IL-1*β* protein from BMDMs was measured by ELISA after treatment with LPS and ATP. ^∗^*p* < 0.05 vs. control, ^†^*p* < 0.05 vs. LPS, ^‡^*p* < 0.05 vs. NCD LPS+ATP, and ^ɤ^*p* < 0.05 vs. HFD LPS+ATP.

## Data Availability

Data and materials have been provided in the sections of methods and results.
